The article "BP Neural Network Based on Simulated Annealing Algorithm Optimization for Financial Crisis Dynamic Early Warning Model" was retracted in 2023. Reasons: suspected computer-generated content; unreliable results or conclusions; concerns about the data; concerns about the results or conclusions.

# BP Neural Network Based on Simulated Annealing Algorithm Optimization for Financial Crisis Dynamic Early Warning Model

**DOI:** 10.1155/2021/4034903

**Published:** 2021-10-07

**Authors:** Ying Chen

**Affiliations:** School of Accounting, Tongling Univesity, Tongling 244000, Anhui, China

## Abstract

Financial early warning mechanism is of great significance to the long-term healthy development and stable operation of listed enterprises. This paper adopts the logistic regression early warning model and BP neural network early warning model. Based on the BP neural network *t* early warning model optimized by the simulated annealing algorithm, the prediction effects of the model are compared from the perspectives of model accuracy and variable importance. Through the comparative analysis of the empirical results of the three methods, it can be seen that the simulated annealing algorithm has many advantages. The combination of the simulated annealing algorithm with multithreading, data compression, and segmentation greatly improves the efficiency of the algorithm and shortens the running time. Using the logistic regression early warning model and BP neural network early warning model and based on the BP neural network *t* early warning model optimized by the simulated annealing algorithm, the prediction effects of the model are compared from the perspective of model accuracy and variable importance. The results show that the three index dimensions of the BP neural network optimized by the simulated annealing algorithm have good discrimination ability to financial status. The BP neural network early warning model optimized based on the simulated annealing algorithm has good prediction accuracy and good practical significance.

## 1. Introduction

The financing demand of high-tech enterprises is huge. Once financial distress occurs, it will not only bring losses to the external stakeholders of the enterprise but also affect the innovation [1]. At present, ST, the risk warning sign of the new third board, is still lagging after the event information. Once ST is marked, financial distress will have a chain effect of deterioration [2]. For investors, creditors, and other external stakeholders, the early warning results of financial distress can be used as the wind vane of investment to help stakeholders monitor the changes of indicators in financial performance, innovation investment, and other aspects of the enterprise, timely discover the potential financial risks of the enterprise, guide investment decisions, and reduce investment risks [3]. Therefore, the construction of the financial early warning mechanism of the new third board is important to the long-term healthy development of the enterprises listed and the stable operation. Therefore, the establishment of financial distress early warning model of high-tech listed enterprises can timely monitor and feedback the financial performance, corporate governance and innovation behavior of high-tech listed enterprises and other indicators, which is conducive to prompt enterprises to timely adjust their decisions and establish a healthy development mechanism.

The article "BP Neural Network Based on Simulated Annealing Algorithm Optimization for Financial Crisis Dynamic Early Warning Model" was retracted in 2023. Reasons: suspected computer-generated content; unreliable results or conclusions; concerns about the data; concerns about the results or conclusions.

The innovation of this paper is to use the logistic regression early warning model and BP neural network early warning model. Based on the BP neural network *t* early warning model optimized by the simulated annealing algorithm, the prediction effects of the model are compared from the perspective of model accuracy and variable importance. Through the comparative analysis of the empirical results of the three methods, it can be seen that the simulated annealing algorithm has many advantages. The combination of the simulated annealing algorithm with multithreading, data compression, and fragmentation greatly improves the efficiency of the algorithm and shortens the running time. At the same time, the simulated annealing algorithm also considers the sparse training data, which is helpful to train the table data with more missing values and provides important value for the research and application of practical problems.

This paper is divided into five sections.  Section 1 presents the background of this study, and Section 2 discusses related work.  Section 3 shows the construction content of the dynamic early warning model.  Section 4 is empirical research.  Section 5 concludes this work.

## 2. Related Work

Chen and Zeng defined the status of a company in financial distress, including bankruptcy, default on debt, and default on preferred stock dividends, and used the cash flow debt ratio index to distinguish its financial status [4]. Shuang et al. initiated the method of using the *Z*-value model to judge the bankruptcy risk of a company, which has important reference value until now [5]. Shuang et al. redefined the definition of financial distress, predicted the probability of financial distress through the financial characteristics of enterprises, and improved the early warning method of financial distress by using the logit model [6]. Dong et al., on the basis of traditional enterprise financial indicators, designed the inventory turnover rate and inventory scale, carried out logistic regression analysis and empirical research on the correlation between inventory risk and financial crisis, and concluded that the inventory turnover rate is inversely proportional to financial crisis, and the inventory scale is directly proportional to financial crisis. The traditional statistical method provides an effective and easy to explain way for the research. With the development of the times, the quantity and quality of enterprise data are constantly improving. At present, more and more data mining and artificial intelligence are applied to the research of early warning [7]. Zhu and Wu established a new risk model by adding three accounting ratio components of three market-driven variables on the basis of the univariate model and confirmed that it is better than the univariate model through classification accuracy and bankruptcy prediction test [8]. Wang et al. used five statistical techniques to predict banks' financial strength ratings (FSRs) [9]. In the aspect of early warning index research, it has experienced the process from the simple financial performance index to comprehensive financial, nonfinancial, and other multidimensional index system. Wang et al., based on the supply basis of accounting information, including indicators reflecting the disclosure of accounting information, taking Shanghai and Shenzhen listed companies as samples, demonstrated that the indicators simplified by the rank sum test can improve the accuracy of the neural network model in predicting financial crisis [10]. Based on the dual perspectives of internal corporate governance and external financial information, Zhang and Yu also included indicators reflecting shareholders, board of directors, management, and board of supervisors and trained the model with SVM, which achieved good prediction results [11]. Wang et al. selected typical indicators of corporate finance and corporate governance, extracted key factors through index difference analysis, factor analysis, and other steps, and carried out SVM analysis of financial early warning of individual corporate financial indicators and SVM analysis of comprehensive financial early warning with corporate governance variables [12]. Yang et al., in the empirical study took cash flow as the key variable, comprehensively considered macroeconomic, monetary policy, and other external factors, established the CFAR model of risk exposure, separated the enterprise expected cash flow and risk cash flow, and used them as the input variable to construct the logistic financial early warning mechanism; the final prediction accuracy reached more than 80% and achieved good model effect [13]. Xu et al. started from the incentive, constraint, and balance mechanism contained in the company's internal governance, selected indicators from the three levels of shareholders, board of directors, and managers, and incorporated them into the financial early warning index system together with the core financial indicators to establish a logistic early warning model. The results of empirical research show that, compared with the traditional financial index model, the model with the introduction of the corporate internal governance index has better discrimination ability, and the performance of the model has been further improved [14]. Zhou et al. expanded the previous bankruptcy index analysis and constructed three kinds of financial early warning models: multiple linear regression, Fisher linear discriminant, and logistic regression to analyze and predict the financial distress of enterprises. Later, scholars' research mainly focused on the improvement of the index system and model method and empirically tested the theoretical model based on different samples of listed companies [15]. Zhang and Huang, based on the essential characteristics of cash flow from operating activities, discussed the relationship between the adequacy, stability, structural rationality and growth of cash flow, and occurrence of financial crisis, selected corresponding indicators from the four characteristics to build a financial early warning system, and established a logistic regression model with other typical financial indicators as control variables. The conclusion shows that the four characteristics are negatively correlated with the probability of financial crisis [16]. Zhang et al., based on the idea of sensors, formed sensor signals through network public opinion analysis, established a financial early warning index system with big data combined with financial indicators, and established a financial early warning model using SVM [17]. The empirical results show that the financial early warning model with big data indicators has better prediction effect than the traditional financial early warning model. On the basis of traditional financial indicators, Hua and Jiang included nonfinancial indicators such as audit opinion and ultimate control human type and, through rough set theory, experienced the process of transition from the traditional statistical method to rapidly change the big data method [18]. On the basis of the support vector machine (SVM), Wang and Zeng used particle swarm optimization (PSO) to optimize feature collection and kernel function at the same time. In this paper, we selected seven indicators of company finance and company size to build an early warning index system. The results of empirical research show that the PSO-SVM model can effectively improve the SVM's ability of early warning of corporate financial crisis [19]. Yao and Wang took Shanghai and Shenzhen *A*-share listed companies as research samples and selected four financial indicators reflecting the debt paying ability, growth ability, profitability, and operating ability of enterprises [20]. The financial early warning model based on the Bayesian discriminant method is established, and good prediction effect is achieved. Song et al., based on the prediction results of the Fisher discriminant analysis model and logistic regression model, established a new nonlinear combination method based on the BP neural network and demonstrated the advantages of the combination prediction model compared with the single prediction model [21]. Sun and Lei started from the idea of interval moderation and integrated the selected financial indicators. The results of empirical research show that the prediction model with the interval index method has high prediction accuracy and clear financial and economic significance [22]. Sun focused on the enterprise's cash flow indicators, selected the financial indicators reflecting the enterprise's operating efficiency, solvency, profitability, and capital gains, and used the classical model, linear probability model, and logistic model for comparative analysis. The empirical research shows that the two models have good prediction effect, and the logistic model has stronger practicability [23]. Chen also used linear regression, linear discrimination, artificial intelligence, and other methods to establish the financial early warning model and demonstrated the superiority of the artificial intelligence method in financial crisis prediction through the comparison of prediction effect between models [24]. Yu et al. broadened the traditional single classifier machine learning method, used AdaBoost (adaptive enhancement algorithm) in boosting to integrate the base classifier support vector machine, increased the weight of error training samples in the training process, and improved the generalization of the model. The results of empirical research show that the performance of the integrated strong classifier is better than that of a single classifier, and it has a higher accuracy in financial early warning [25].

The article "BP Neural Network Based on Simulated Annealing Algorithm Optimization for Financial Crisis Dynamic Early Warning Model" was retracted in 2023. Reasons: suspected computer-generated content; unreliable results or conclusions; concerns about the data; concerns about the results or conclusions.

Throughout the research on financial distress early warning in recent years, it is found that most scholars use early warning indicators with similar dimensions, combined with artificial intelligence comprehensive models such as univariate decision-making model, multivariate discriminant model, logistic regression model, neural network model, and support vector machine model. Different models have different early warning effects. Generally speaking, there is still much room for improvement and exploration in the research of financial distress early warning, which is mainly reflected in the following three aspects: (1) most of the existing financial distress early warning research is focused on the main board listed companies, while there is less research on the new third board listed companies, especially for specific industries with common characteristics. (2) There are few studies on nonfinancial factors. For small- and medium-sized high-tech enterprises, the performance of nonfinancial indicators reflecting the dimension of innovation behavior, such as investment proportion, cannot be ignored. They can be considered to be included in the financial early warning system. The existing early warning model methods still have room for further development, such as simulated annealing algorithm and other integrated classifier methods, which have good error control and generalization ability. It also has certain research and application value.

## 3. Construction of Dynamic Early Warning Model

This paper uses the logistic regression early warning model and BP neural network early warning model. Using the logistic regression early warning model and BP neural network early warning model, based on the BP neural network warning model optimized by the simulated annealing algorithm, the prediction effects of the model are compared from the perspective of model accuracy and variable importance. Construction of the BP neural network dynamic early warning model BP neural network model includes the following aspects.

The BP neural network model includes

(1) Model and parameters: the linear model is a typical example [26, 27]. The output variable prediction formula of the linear model is ${\hat{y}}_{i}=\sum_{j}\theta_{j}x_{ij}$, and its essence is the linear combination of weighted input variable characteristics. Depending on the attributes of the model classification or regression, the predicted values can have different interpretations. For example, in the classification mode, it can carry out logical transformation to obtain classification in the logical regression. In the regression model, the expected values of numerical variables can be obtained.
Parameters refer to the undetermined parts that need to be determined through machine learning of data. In the linear regression problem, the parameter is the coefficient *θ*. The Greek letter *θ* is usually used to represent parameters in the model.
(2) Objective function: the remarkable feature of the objective function is that it consists of training loss and regularization: objective function = training loss + regularization, as shown in the following formula:
  (1) $$\begin{array}{c} \text{obj}\left(\theta \right)=L\left(\theta \right)+\Omega \left(\theta \right). \end{array}$$
The raining loss*L*can be used to measure the influence of the model on training times.

According to the data, it can be predicted. The common choice is the mean square error, as shown in the following formula:

(2) $$\begin{array}{c} L\left(\theta \right)=\sum_{i}{\left(y_{i}-{\hat{y}}_{i}\right)}^{2}. \end{array}$$

Another common loss function is the logical loss for logistic regression, which is given by the following formula:

(3) $$\begin{array}{c} L\left(\theta \right)=\sum_{i}\left[y_{i}\ln\left(1+e^{-{\hat{y}}_{i}}\right)+\left(1-y_{i}\right)\ln\left(1+e^{{\hat{y}}_{i}}\right)\right]. \end{array}$$

The regular term is a part that is often missed. It can control the complexity of the model and effectively avoid overfitting.

The article "BP Neural Network Based on Simulated Annealing Algorithm Optimization for Financial Crisis Dynamic Early Warning Model" was retracted in 2023. Reasons: suspected computer-generated content; unreliable results or conclusions; concerns about the data; concerns about the results or conclusions.

The principle of equilibrium between objective functions is to train a model with simplicity and predictability at the same time. The trade-off between the two is also called deviation variance trade-off.

The model selection of the simulated annealing algorithm is decision tree set. Usually, the strength of a single tree is not enough to be used in practice. The actual use is the ensemble model, which adds the predictions. Mathematical model formula (4) of multiple trees complement each other:

(4) $$\begin{array}{c} {\hat{y}}_{i}=\sum_{k=1}^{K}f_{k}\left(x_{i}\right),\;f_{k}\in F. \end{array}$$

Specifically, *f*(*x*)=*w*_*q*(*x*)_ represents the regression decision tree learner, *q* represents the leaf index corresponding to the structure of each tree, and *q*(*x*) ∈ {1,2,3,…, *T*}, where *T* represents the number of leaf nodes. Different from the GBDT model, the regularization term is added to the objective function of the simulated annealing algorithm:

(5) $$\begin{array}{c} \text{obj}\left(\theta \right)=\sum_{i}^{n}l\left(y_{i},{\hat{y}}_{i}\right)+\sum_{k=1}^{K}\Omega \left(f_{k}\right), \end{array}$$

where *l* in the above formula represents the differentiable convex loss function, which is used to measure the difference between the predicted value $\hat{y}$ and the actual value *y*_*i*_.(such as regression tree function). This additional conventional term can help smooth the final learning weight of the model to avoid overfitting. EE represents the complexity penalty term of the model. According to the relevant definitions of the regression tree, the regular term function can be expressed as the following formula:

(6) $$\begin{array}{c} \Omega \left(f\right)=\gamma T+\frac{1}{2}\lambda {\left\|w\right\|}^{2}. \end{array}$$

The addition of the regular term reflects the principle that models tend to choose models with both simplicity and predictability. The model returns to the traditional GBDT model.

The article "BP Neural Network Based on Simulated Annealing Algorithm Optimization for Financial Crisis Dynamic Early Warning Model" was retracted in 2023. Reasons: suspected computer-generated content; unreliable results or conclusions; concerns about the data; concerns about the results or conclusions.

An additional method, namely, iterative method, is used to train the model. Let ${\hat{y}}_{i}^{\left(t\right)}$ be the prediction of the *i* instance by the model in the *t* iteration, and the iterative updating method is shown in the following formula:

(7) $$\begin{array}{c} {\hat{y}}_{i}^{\left(t\right)}=\sum_{k=1}^{t}f_{k}\left(x_{i}\right)=y_{i}^{\left(t-1\right)}+f_{t}\left(x_{i}\right). \end{array}$$

Further, the objective function becomes

(8) $$\begin{array}{c} {\text{obj}}^{\left(t\right)}=\sum_{i=1}^{N}l\left(y_{i},{\hat{y}}_{i}^{\left(t\right)}\right)+\sum_{i=1}^{t}\Omega \left(f_{i}\right)=\sum_{i=1}^{N}l\left(y_{i},{\hat{y}}_{i}^{\left(t-1\right)}+f_{t}\left(x_{i}\right)\right)+\Omega \left(f_{\text{t}}\right). \end{array}$$

For any form of the loss function, the second-order Taylor expansion approximation method can be used to achieve fast optimization, such as the following formula:

(9) $$\begin{array}{c} {\text{obj}}^{\left(t\right)}=\sum_{i=1}^{N}{}_{\sum }^{N}\left[l\left(y_{i},{\hat{y}}_{i}^{\left(t-1\right)}+g_{i}f_{t}\left(x_{i}\right)\right)+\frac{1}{2}h_{i}f_{i}^{2}\left(x_{i}\right)\right]+\Omega \left(f_{\text{t}}\right), \end{array}$$

where *g*_*i*_ and *h*_*i*_ represent the first-order and second-order gradient statistics of the loss function, respectively, as shown in the following formula:

(10) $$\begin{array}{c} g_{i}=\partial_{{\hat{y}}_{i}^{\left(t-1\right)}}l\left(y_{i},{\hat{y}}_{i}^{\left(t-1\right)}\right),\\ h_{i}=\partial_{{\hat{y}}_{i}^{\left(t-1\right)}}^{2}l\left(y_{i},{\hat{y}}_{i}^{\left(t-1\right)}\right). \end{array}$$

After the constant term is removed, the reduced objective function of the *t*th iteration is obtained, as shown in the following formula:

(11) $$\begin{array}{c} {\text{obj}}^{\left(t\right)}=\sum_{i=1}^{N}\left[g_{i}f_{t}\left(x_{i}\right)+\frac{1}{2}h_{i}f_{i}^{2}\left(x_{i}\right)\right]+\Omega \left(f_{\text{t}}\right). \end{array}$$

It can be seen that the simulated annealing algorithm only needs to add the first order, which greatly reduces the dependence of the model.

After substituting into the penalty function, *I*_*i*_={*i|q*(*x*_*i*_)=*j*} is defined, and the objective function is further changed into the following formula:

(12) $$\begin{array}{c} {\text{obj}}^{\left(t\right)}=\sum_{i=1}^{N}\left[g_{i}f_{t}\left(x_{i}\right)+\frac{1}{2}h_{i}f_{i}^{2}\left(x_{i}\right)\right]+\gamma T+\frac{1}{2}\lambda \sum_{j=1}^{T}w_{j}^{2}=\sum_{i=1}^{N}\left[\left(\sum_{i\in I_{i}}g_{i}\right)w_{j}+\frac{1}{2}\left(\sum_{i\in I_{i}}h_{i}+\lambda \right)w_{j}^{2}\right]+\gamma T. \end{array}$$

For a fixed structure *q*(*x*), the best predictive value *w*_*j*_^*∗*^ corresponding to the *j* leaf node can be calculated, namely, the following formula:

(13) $$\begin{array}{c} w_{j}^{*}=-\frac{\sum_{i\in I_{i}}g_{i}}{\sum_{i\in I_{i}}h_{i}+\lambda }. \end{array}$$

At the same time, the corresponding optimal objective function value can be calculated, namely, the following formula:

(14) $$\begin{array}{c} {\text{obj}}^{*}=-\frac{1}{2}\sum_{j=1}^{T}\frac{{\left(\sum_{i\in I_{i}}g_{i}\right)}^{2}}{\sum_{i\in I_{i}}h_{i}+\lambda }+\gamma T. \end{array}$$

Formula (14) is similar to the impure evaluation of the decision tree, but it comes from a broader objective function.

The article "BP Neural Network Based on Simulated Annealing Algorithm Optimization for Financial Crisis Dynamic Early Warning Model" was retracted in 2023. Reasons: suspected computer-generated content; unreliable results or conclusions; concerns about the data; concerns about the results or conclusions.

In general, starting from the root node, iteratively adding branches to the tree based on some node classification rules to form the best decision tree. Formula (15) is often used to determine candidate splitting nodes in practice:

(15) $$\begin{array}{c} L_{\text{split}}=\frac{1}{2}\left[\frac{{\left(\sum_{i\in I_{R}}g_{i}\right)}^{2}}{\sum_{i\in I_{R}}h_{i}+\lambda }+\frac{{\left(\sum_{i\in I_{L}}g_{i}\right)}^{2}}{\sum_{i\in I_{L}}h_{i}+\lambda }-\frac{{\left(\sum_{i\in I}g_{i}\right)}^{2}}{\sum_{i\in I}h_{i}+\lambda }\right]-\gamma . \end{array}$$

The above formula consists of four parts: new left lobe score, new right lobe score, original lobe score, and regular term. When the gain is less than *γ*, that is, *L*_split_ < 0, it is proved that the information gain caused by node splitting is not enough to make up for the complexity penalty loss caused by increasing leaf nodes. At this time, the model chooses not to add branches, which is similar to the prepruning technology in the decision tree model, as shown in Figure 1.

To sum up, the model optimized greatly improves the performance of the prediction model, and its specific advantages include the following: (1) regularization lifting technology can effectively help the model reduce the over fitting problem. (2) Parallel processing of feature granularity greatly improves the speed of model training. (3) The optimization objectives and evaluation criteria are flexible. (4) Perfect missing value processing rules. (5) After splitting to the maximum depth, pruning can avoid ignoring the comprehensive positive loss. (6) Built-in cross validation is used to obtain the optimal number of iterations. (7) We can continue to train on the basis of the existing model. The simulated annealing algorithm finds the best splitting mode quickly and effectively by traversing the candidate splitting nodes and optimizing the traversal order by presorting.

## 4. Empirical Research

This paper constructs the financial distress early warning model. The parameters of the network model optimized by the simulated annealing algorithm include conventional parameters, lifter parameters, and task parameters. Conventional parameters mainly control the macrofunction. The research goal of this paper is the financial distress early warning two-classification problem; let the booster be gbtree and train samples based on tree model. The elevator parameters are used to control the tree model of each step. ETA shrinkage step size, namely, learning rate, can prevent overfitting problem. By reducing the weight of features, the lifting calculation process is more conservative and the robustness of the model is improved. max_depth represents the maximum depth of each tree. If the depth is too large, it will easily lead to overfitting. If the depth is too small, it may lead to insufficient learning. Compared with the benchmark model, the model algorithm proposed in this paper can prevent the overfitting problem. By reducing the weight of features, the calculation process is more conservative and the robustness of the model is improved. Min_ child_ weight parameter determines the sample weight sum of the minimum leaf node, which is used to avoid learning local special samples, but too high value will lead to underfitting. The Gamma parameter, with a default value of 0, specifies the minimum drop in the loss function required for a leaf node to continue splitting. The larger the setting value is, the more conservative the algorithm is. The subsample parameter controls the proportion of random sampling for each tree. Task parameters determine the ideal optimization goal and the measurement method of each step result. Objective defines the type of minimization loss function. It defines the parameter as binary: logistic binary logistic regression model to return the prediction probability value.

The article "BP Neural Network Based on Simulated Annealing Algorithm Optimization for Financial Crisis Dynamic Early Warning Model" was retracted in 2023. Reasons: suspected computer-generated content; unreliable results or conclusions; concerns about the data; concerns about the results or conclusions.

Because the judgment of financial distress in this paper is a two-classification problem [28–30], the loss function is determined as “c e” interactive entropy. Ten-fold cross-validation method is used to train data, and BP neural network models are established for T-2 and T-3 data, respectively. The structure diagram of the BP neural network model optimized by the simulated annealing algorithm is shown in Figure 2. The training results show that 11515 iterations have been carried out in T-2, and the loss function is 203.36. A total of 1385 iterations were carried out in T-3, and the loss function was 108.26.

### 4.1. Model Prediction

From Table 1, the average accuracy rates of T-2 and T-3 BP neural network optimized based on the simulated annealing algorithm for financial distress early warning are 88.16% and 77.34%, respectively, and the optimal accuracy rates are 90.10% and 80.00%, respectively. The discrimination ability of actual distress enterprises is enhanced. This shows that the BP neural network model has good fault tolerance and generalization ability. At the same time, the prediction accuracy of T-2 is still higher than that of T-3, which further proves that, with the approaching of the year of financial distress, the discrimination of indicators is significantly enhanced.

The article "BP Neural Network Based on Simulated Annealing Algorithm Optimization for Financial Crisis Dynamic Early Warning Model" was retracted in 2023. Reasons: suspected computer-generated content; unreliable results or conclusions; concerns about the data; concerns about the results or conclusions.

In order to intuitively compare the importance of seven input variables for financial distress or health status discrimination, R software was used to draw the generalized weight scatter diagram of seven input variables and their factors at each observation point. The ordinate GVV represents the generalized weight, and the abscissa represents the observed value. The generalized weighted scatter plots of T-2 and T-3 are shown in Figures 3 and 4, respectively. The importance of seven input variables in different prediction periods can be compared by the observation concentration in the generalized weighted scatter diagram. As can be seen from Figures 3 and 5, in T-2, the observation generalized weights of the three factors of F2 innovation profitability, F4 operation capability, and F6 growth capability are mostly concentrated around 0, indicating that these three factors have relatively little effect on judging financial distress or health status, while F1 business profitability, F3 solvency, F5 capital structure, and F7 equity structure are relatively important and show a certain nonlinear relationship. When the forecast period is advanced to T-3 years, it can be found that the importance of the seven input variables is weakened, and the observation generalized weights tend to concentrate around 0. However, in comparison, the F3 solvency factor and F5 capital structure factor are more important, and the observation generalized weights are more dispersed. It shows that these two factors have strong long-term influence and better performance in long-term prediction.

Output of the importance results of T-2 and T-3 model training characteristic variables is shown in Figure 4.

As can be seen from Figure 4, in the T-2 financial distress early warning model, the F7 equity structure factor accounts for more than 0.4, which is the most important factor, and F3 operating capacity factor accounts for more than 0.3, which is the second important factor, followed by the F5 capital structure factor, F6 growth capacity factor, F4 solvency factor, F1 business profitability factor, and F2 innovation profitability factor. The importance of these five factors is less than 0.1. Therefore, in the T-2 financial distress early warning model, the F7 ownership structure factor and F3 operating capacity factor are the key variables to judge whether the company will fall into financial distress.

The article "BP Neural Network Based on Simulated Annealing Algorithm Optimization for Financial Crisis Dynamic Early Warning Model" was retracted in 2023. Reasons: suspected computer-generated content; unreliable results or conclusions; concerns about the data; concerns about the results or conclusions.

The forecast time is one year ahead of schedule. In the T-3 early warning model, the importance of early warning indicators has changed. The importance of the F1 business profitability factor, F5 capital structure factor, F3 operating capacity factor, and F7 equity structure factor is more than 0.1, of which the proportion of the F1 business profitability factor is more than 0.3, and the proportion of F5 capital structure factor is more than 0.2.

Generally speaking, in the two-stage simulated annealing algorithm financial distress early warning model, the F1 business profitability factor, F3 operating capacity factor, F5 capital structure factor, and F7 equity structure factor have a greater contribution to the model prediction and have a better long-term prediction ability. From the perspective of practical significance, enterprises should strengthen the management performance, debt ability, equity system, and other aspects of management and control, in order to avoid the occurrence of financial difficulties.

After completing the training and test set evaluation of the above basic model, the AUC value obtained in the evaluation process can be used as the AUC benchmark value in feature contribution analysis. In order to get the contribution of each feature, this paper uses the shuffling algorithm to shuffle each feature data in the test set randomly and obtains 6749 new test sets corresponding to each feature. After using the basic model to classify them, we can get the new AUC value after shuffling the test set features. Finally, this paper uses the absolute value of the change of AUC relative to the benchmark AUC after feature shuffling as the index of feature contribution. The contribution degree of feature f1-f6745 is calculated, as shown in Figure 6. From the figure, it is known that the contribution of each feature to the model is relatively concentrated on the whole. But the contribution of some features is obviously high or low. Extracting these features with high or low contribution may be helpful to the development of business. The absolute value also shows that the basis of model judgment is usually not a single feature, but a complex combination of features.

#### 4.1.1. Comparison of Model Results

Based on T-2 and T-3 years' early warning index data, this paper establishes logistic regression and simulated annealing algorithm, respectively, and compares and evaluates the performance of the models from the perspectives of prediction accuracy and variable importance.

In order to further compare the performance of the models used in this paper, this paper trains some other commonly used classifiers based on the same training set, uses them to complete the classification of the test set, and compares the characteristics of each model from the index. When choosing other models as the comparison reference, this paper mainly includes the linear model, support vector machine model using Gaussian kernel function, and tree model.  Figure 7 shows the ROC curve of each model for the test set classification results. In addition to logistic regression, the ROC curves of other models are in a relatively concentrated position, with a little overlap, indicating that there are some differences in AUC indicators, but the overall difference is not big, so it is necessary to further analyze the advantages and disadvantages of each model combined with other indicators.

The article "BP Neural Network Based on Simulated Annealing Algorithm Optimization for Financial Crisis Dynamic Early Warning Model" was retracted in 2023. Reasons: suspected computer-generated content; unreliable results or conclusions; concerns about the data; concerns about the results or conclusions.

First of all, from the perspective of the accuracy of the early warning model, the early warning accuracy of the simulated annealing algorithm is higher than the other two models in both the T-2 and T-3 periods. At the same time, it can be seen that the closer the time from the occurrence of financial distress, the better the prediction effect of the model, which reflects that financial distress is a gradual process, and the closer the time, the indicators have greater differences and more sensitive causality. For the internal and external stakeholders of the enterprise, the forecast results with larger time interval can provide longer adjustment time. On the one hand, it is helpful for the operators to timely adjust the business direction, innovation investment, and other strategic decisions. On the other hand, it is helpful for the investors to better grasp the financial dynamics of the investment object and guide the investment portfolio.

Secondly, from the explanatory point of view of the model, the three models can compare the importance of variables. The logistic regression model is more intuitive for the expression of the significance of variables, and the economic significance of the model is strong. The important results of the variables of the three types of early warning models are basically consistent, that is, the variables of F1 business profitability, F3 solvency, F5 capital structure, and F7 equity structure have a greater impact on the identification of financial distress or health status, and F5 capital structure has a better long-term forecasting ability. Finally, from the perspective of the operation speed and time efficiency of the model, the simulated annealing algorithm has faster training speed, which is significantly better than the other two models. The results of the comparison of the three models are shown in Figure 8.

The article "BP Neural Network Based on Simulated Annealing Algorithm Optimization for Financial Crisis Dynamic Early Warning Model" was retracted in 2023. Reasons: suspected computer-generated content; unreliable results or conclusions; concerns about the data; concerns about the results or conclusions.

## 5. Conclusion

Through the comparative analysis of the empirical results of the three methods, we can see that the simulated annealing algorithm has many advantages. The simulated annealing algorithm combined with multithreading, data compression and fragmentation greatly improves the efficiency of the algorithm and shortens the running time. At the same time, the simulated annealing algorithm also considers the case that the training data is sparse, which helps to train the table data with more missing values, and provides important value for the research and application of practical problems, especially in the economic and social fields. Therefore, considering the financial distress early warning for high accuracy and strong explanatory requirements, the simulated annealing algorithm with superior generalization ability and error control ability can achieve better practicability.

## Figures and Tables

**Figure 1:** Flowchart of the BP neural network model optimized by the simulated annealing algorithm.

**Figure 2:** A BP neural network flowchart optimized by a simulated annealing algorithm based on dynamic financial early warning classification.

**Figure 3:** The T-3-year generalized weight scatter diagram.

**Figure 4:** Importance comparison of T-2 (a) and T-3 (b) variables.

**Figure 5:** The T-2-year generalized weight scatter diagram.

**Figure 6:** Contribution degree of individual characteristics.

**Figure 7:** Three model ROC values.

**Figure 8:** Comparison of the three models.

**Table 1:** Classification table of prediction results of the BP neural network early warning model.

			Actual category		Optimal/average accuracy
			Healthy 0	Dilemma 1	
T-2	Forecast category	Healthy 0	78	10	—
		Dilemma 1	0	13	
Optimal accuracy/average accuracy					90.10%/88.16%

T-3	Forecast category	Healthy 0	24	8	—
		Dilemma 1	1	12	
Optimal/average accuracy					80.00%/77.34%

## Data Availability

The data used to support the findings of this study are available from the corresponding author upon request.
